This article has been retracted.

# Use of biologics in patients with psoriasis – A retrospective analysis based on real‐world data

**DOI:** 10.1111/srt.13550

**Published:** 2024-01-04

**Authors:** Jing Pan, Xiaodan Chang, Lingyan Wang, Gang Miao, Qiuzi Jin, Ningning Guo, Jiayu Zhang, Yanwei Lv, Lifang Wang

**Affiliations:** ^1^ Department of Dermatology and Venereology Beijing Jishuitan Hospital, Capital Medical University Beijing China; ^2^ National Clinical Research Center for Dermotologic Diseases and Immunologic Diseases Beijing China; ^3^ Department of Clinical Epidemiology Research Center Beijing Jishuitan Hospital, Capital Medical University Beijing China

**Keywords:** biologic agents, PASI, psoriasis, real world research, secukinumab

## Abstract

**Objective:**

To summarize and analysis the application of biologic agents in patients with psoriasis in the real world.

**Methods:**

Relying on collected data from June 2020 to September 2021 in the database of China Psoriasis Standardized Diagnosis and Treatment Center, 2529 cases of psoriasis patients treated with biologic agents in 188 different tertiary hospitals across China were retrospective analyzed. The collected information mainly includes demographic data (age, gender, psoriasis history), curative effectiveness of used biologics drug withdrawal and its reason. According to the collected information, condition of the usage for each category of biologics and influencing factor of biologics replacement were analyzed.

**Result:**

A total of 2529 patients were analyzed, which included 1626 male (64.29%) and 903 female (35.71%) with an average age of 42.12 ± 14.70 (17 ∼ 85) years old; 2336 (92.37%) patients were aged from 19 to 60 years old. Within these patients, 2362 of them (93.40%) had a psoriasis area and severity index (PASI) score, and 1776 of these patients had moderate to severe cases (75.19%). According to the patient's self‐evaluation of the past efficacy of biological agents, secukinumab was chosen by the most people to have the highest efficacy (1140 cases, 93.60%). The main reason for the withdrawal of secukinumab is that the disease is already well controlled at the time of withdrawal (67 cases, 38.95%); for TNF‐ α inhibitor is the poor curative effect; for ustekinumab and ixekizumab were the non‐affordable price.

**Conclusions:**

In the current biotherapy of psoriasis in China, the efficacy of secukinumab is thought by most people to be the highest. Secukinumab is the first choice when the needs of changing biologics appear.

## 1 INTRODUCTION

In recent years, biologics for the treatment of psoriasis have been developing rapidly, with particularly favorable efficacy achieved for the treatment of moderate to severe, refractory and special types of psoriasis. China's National Medical Products Administration has approved the following two categories of biologics for the treatment of psoriasis: (1) tumor necrosis factor (TNF)‐α inhibitors, including etanercept, infliximab, and adalimumab; and (2) interleukin inhibitors, including ustekinumab, secukinumab, ixekizumab, and guselkulmab. In addition, more biologics are currently being developed. The data used in this study were sourced from the Database of Chinese Center for Standardized Diagnosis and Treatment of Psoriasis, which is the first nationwide collaborative program initiated by the National Clinical Research Center for Dermatologic and Immunologic Diseases (supported by Department of Dermatology, Peking University First Hospital) in August 2020. Statistical analyses were performed on the real‐world clinical data of 2529 psoriasis patients treated with biologics collected from June 2020 to September 2021 from various perspectives, including the proportions of patients using different biologics, differences in the selection of biologics in patients with different types of psoriasis, the efficacy of different biologics, and the factors affecting drug discontinuation, and the current status of the use of biologics in China is summarized, in an effort to provide evidence for clinicians in using biologics to treat psoriasis.

## 2 SUBJECTS AND METHODS

### 2.1 Subjects

About 2529 psoriasis patients treated with biologics (1049 of which had follow‐up records) included in the Database of Chinese Center for Standardized Diagnosis and Treatment of Psoriasis from June 2020 to September 2021 were collected retrospectively. These patients were from 188 tertiary hospitals in 44 cities in 16 provinces across China, and all the data were desensitized. All patients signed an Informed Consent Form when entering the database, and this study was approved by the Medical Ethics Committee of Beijing Jishuitan Hospital (approval number: JiLunKeShenZi No.202109‐57). Inclusion criteria: (1) clinical diagnosis of psoriasis; (2) any age and gender; (3) prior use of biologics or starting to use biologics when entering the database; (4) patients with follow‐up records; (5) patients with adverse reaction records. Exclusion criteria: (1) incomplete essential patient data; (2) medication history unknown or history of using other drugs contraindicated for concomitant use of biologics; (3) other co‐morbidities that may affect treatment, for example, autoimmune diseases, tumors, HIV infection, uncontrolled hypertension, and cardiac insufficiency.

### 2.2 Data collection

The patients’ demographics (age, gender, medical history), psoriasis classification, types of biologics used, efficacy, whether discontinued drug and reasons for discontinuation, and whether changed biotherapy regimen, etc., were primarily collected. Prior efficacy was evaluated based on the patient self‐rated outcomes in the system, including good, average, or poor. Age was classified by the age groups of 0–18, 19–44, 45–60, and ≥61 years for analysis as categorical statistics. The Psoriasis Area and Severity Index (PASI) was used to evaluate the severity of psoriasis, where a score of <3 would be classified as mild, a score of 3–9 as moderate, and a score of ≥10 as severe.

### 2.3 Quality control

The collected data were subjected to logic check and proof‐checking for completeness. A total of 2599 pieces of data were collected in this study. After excluding 61 pieces of data with more than three empty entries and nine pieces of data with logical errors, a total of 2529 pieces of data (involving 2529 patients) were included in the analysis of this study.

### 2.4 Statistical methods

Statistical analysis was performed using SPSS 26.0. Normality analysis of statistics was performed using Shapiro‐Wilk test. Normally distributed continuous variables were presented as mean ± standard deviation $\left(\bar{x}\pm \cdot s\right)$, comparison between groups were performed using ANOVA, and Least Significant Difference (LSD) method was used for pairwise comparisons; non‐normally distributed continuous variables were described using minimum, maximum, quartiles, and median, and non‐parametric Kolmogorov‐Smirnov method was used for pairwise comparisons. Categorical variables were statistically described using the number or percentage of patients, and chi‐square test was used for pairwise comparisons. *P* < 0.05 would indicate a statistically significant difference.

## 3 RESULTS

### 3.1 General data of patients

Among the 2529 psoriasis patients treated with biologics, 1626 (64.29%) were male, and 903 (35.71%) were female. The age was 42.12 ± 14.70 (17–85) years old; specifically, 45 patients were aged 0–18 years (1.78%), 1508 (59.63%) 19–44 years, 828 (32.74%) 45–60 years, 148 (5.85%) ≥61 years, and 2,336 (92.37%) 19–60 years. The length of psoriasis history was 6 (2, 13) years.

### 3.2 Disease characteristics and application status of biologics in patients with psoriasis

#### 3.2.1 Disease severity in patients of different age groups

Among the 2529 patients, 2362 (93.40%) had a PASI score of 6.60 (2.90, 14.30). There were statistically significant differences in disease severity and PASI score across patients in different age groups (both *P* < 0.001), as presented in Table 1. LSD comparisons showed that the disease severity and PASI score were significantly lower in 0–18 years group than in 45–60 (*P* = 0.011, 0.013) and ≥61 (*P* = 0.048, 0.006) years groups; the disease severity and PASI score were significantly lower in 19–44 years group than in 45–60 years group (both *P* < 0.001), and the PASI score was significantly lower in 19–44 years group than in ≥61 years group (*P* < 0.001), yet was no statistically significant difference between 19–44 years group and ≥61 years group in disease severity (*P* = 0.052); in addition, there were no statistically significant differences in disease severity or PASI score between 0–18 years and 19–44 years groups or between 45–60 years and ≥61 years groups (all *P* > 0.05). Overall, there were 1776 (75.19%) patients with moderate to severe disease, consisting of the majority of patients.

**TABLE 1:** Disease severity in 2362a psoriasis patients of different age groups treated with biologics [*N* (%) or *M* (Q1, Q3)].

		Disease severity			
Age group (years)	*N* patients	Mild (<3 points)	Moderate (3–9 points)	Severe (≥10 points)	PASI score (points)
0–18	45	17(37.78)	16(35.56)	12(26.67)	4.10 (1.80, 10.80)
19–44	1411	404(28.63)	515(36.50)	492(34.87)	5.90 (2.50, 12.70)
45–60	778	143(18.38)	283(36.38)	352(45.24)	8.05 (3.60, 16.78)
≥61	128	22(17.18)	51(39.84)	55(42.97)	8.85 (3.90, 15.60)
Total	2362^a^	586(24.81)	865(36.62)	911(38.57)	6.60(2.90,14.30)
*H* value/chi‐square value		41.24			52.11
*P* value		<0.001			<0.001

*Note*: PASI: psoriasis area and severity index.

^a^ After excluding 167 patients with missing PASI data from 2529 psoriasis patients.

#### 3.2.2 Application status of biologics in patients with different types of psoriasis

Among the 2529 patients, psoriasis vulgaris with plaques as the primary clinical manifestation accounted for the highest proportion of patients (2006, 79.79%), followed by psoriasis vulgaris primarily manifested as guttate lesions (295, 11.73%), erythrodermic psoriasis (75, 2.98%), arthritic psoriasis (74, 2.94%), generalized pustular type (33, 1.31%), and localized pustular type (31, 1.23%). The name of the biologic used was not documented for 15 of the 2529 patients; in reviewing the remaining 2514 patients, 42 patients were found to have been treated with two biologics, so that a total of 2556 patients were considered to have used biologics. Among patients with different psoriasis types, the highest proportion used secukinumab, followed by adalimumab. See Table 2.

**TABLE 2:** Use of biologics in 514 patients with different types of psoriasis [*N* (%)].

			TNF‐α inhibitorsb				Interleukin inhibitorsb			
Psoriasis classification		*N* patients (2514a)	Adalimumab	Etanercept	TNF receptor ‐antibody fusion protein	Infliximab	Ustekinumab	Secukinumab	Ixekizumab	Guselkumab
Vulgaris	Patchy	2006	443(21.75)	40(1.96)	122(5.99)	91(4.47)	25(1.23)	1204(59.11)	99(4.86)	13(0.64)
	Guttate	295	67(21.90)	4(1.31)	25(8.17)	11(3.59)	5(1.63)	183(59.80)	11(3.59)	0(0)
Erythrodermic		75	17(22.67)	2(2.67)	4(5.33)	1(1.33)	0(0)	42(56.00)	9(12.00)	0(0)
Arthritic		74	22(29.73)	0(0)	2(2.70)	2(2.70)	0(0)	44(59.46)	3(4.05)	1(1.35)
Pustular	Generalized	33	11(33.33)	1(3.03)	2(6.06)	3(9.09)	0(0)	13(39.39)	3(9.09)	0(0)
	Localized	31	5(16.13)	1(3.23)	2(6.45)	0(0)	0(0)	22(70.97)	1(3.23)	0(0)

*Note*: a The name of the biologic used was not documented for 15 of the 2529 patients, so that use of biologics was analyzed for the remaining 2514 patients; b42 patients successively used 2 biologics, so that a total of 2,556 patients were counted and included in the table.

#### 3.2.3 Prior efficacy of biologics

Among the 2529 patients, 2144 were evaluated for efficacy of previously used biologics. Based on the patients' self‐rated efficacy of previously used biologics, statistical analysis showed statistically significant difference in efficacy across various previously used biologics (*P* < 0.001). Among all the biologics, secukinumab had the best evaluation of prior efficacy, with 93.60% patients rating it as good, 1.23% rating it as poor, which is the lowest among all biologics, and 5.17% rating it as average. See Table 3.

**TABLE 3:** Comparison of patient self‐rated prior efficacy of different biologics among 2144a psoriasis patients [*N* (%)].

Class of biologics		*N* patients	Prior efficacy		
			Good	Average	Poor
TNF‐α inhibitors	Adalimumab	503	323(64.21)	126(25.05)	54(10.74)
	Etanercept	46	21(45.65)	17(36.96)	8(17.39)
	TNF receptor‐antibody fusion protein	130	38(29.23)	61(46.92)	31(23.85)
	Infliximab	95	54(56.84)	33(34.74)	8(8.42)
Interleukin inhibitors	Ustekinumab	22	18(81.82)	3(13.64)	1(4.55)
	Secukinumab	1218	1140(93.60)	63(5.17)	15(1.23)
	Ixekizumab	116	94(81.03)	17(14.66)	5(4.31)
	Guselkumab	14	13(92.86)	1(7.14)	0(0)
Chi‐square value			488.39		
*P* value			<0.001		

*Note* : ^a^Efficacy evaluation for previously used biologics was performed for a total of 2144 of the 2529 patients.

#### 3.2.4 Reasons for discontinuation of biologics

Among the 2529 patients, a total of 603 discontinued the drug for various reasons, including poor efficacy, safety and tolerability issues, discontinuation after disease control, and economic reasons, etc., as specified in Table 4. The primary reason for discontinuation was discontinuation after disease control for secukinumab (67, 38.95%); poor efficacy for adalimumab (83, 38.43%), etanercept (18, 58.06%), TNF receptor‐antibody fusion protein (39, 44.32%), and infliximab (16, 27.12%); and economic reasons for ustekinumab (2/6) and ixekizumab (8, 29.63%). Other reasons for drug discontinuation include the impact of COVID‐19, personal schedule, ineffectiveness in later stage of use, impact on intelligence, pregnancy, heavy financial burden, and switch to similar drugs covered by medical insurance, etc. Among the patients who discontinued the drug for safety and tolerability reasons, a 49‐year‐old female patient with plaque psoriasis had a baseline PASI score of 0.9 when entering the database and no prior comorbidities such as old pulmonary tuberculosis, yet turned positive for tuberculosis test 2 months into treatment with secukinumab, for which the drug was discontinued; a 20‐year‐old male patient had a baseline PASI score of 26.7 and no prior comorbidities such as viral hepatitis, yet was tested positive for hepatitis B virus antigen 6 months into treatment with ixekizumab, for which the drug was discontinued.

**TABLE 4:** Reasons for discontinuation of biologics in 603 patients [*N* (%)].

			Reason for discontinuation				
Class of biologics		*N* patients	Poor efficacy	Safety and tolerability issues	Discontinuation after disease control	Economic reasons	Other^a^
TNF‐α inhibitors	Adalimumab	216	83(38.43)	35(16.20)	68(31.48)	12(5.56)	18(8.33)
	Etanercept	31	18(58.06)	5(16.13)	5(16.13)	1(3.23)	2(6.45)
	TNF receptor‐antibody fusion protein	88	39(44.32)	11(12.50)	28(31.82)	6(6.82)	4(4.55)
	Infliximab	59	16(27.12)	16(27.12)	13(22.03)	3(5.08)	11(18.64)
Interleukin inhibitors	Ustekinumab	6	1(16.67)	0(0)	1(16.67)	2(33.33)	2(33.33)
	Secukinumab	172	20(11.63)	21(12.21)	67(38.95)	29(16.86)	35(20.34)
	Ixekizumab	27	8(29.63)	3(11.11)	5(18.52)	8(29.63)	3(11.11)
	Guselkumab	4	0(0)	0(0)	3(75.00)	1(25.00)	0(0)

*Note*: ^a^Other reasons for drug discontinuation include impact of COVID‐19, personal schedule, ineffectiveness in later stage of use, impact on intelligence, pregnancy, heavy financial burden, and switch to similar drugs covered by medical insurance, etc.

## 4 DISCUSSIONS

Psoriasis is a chronic immune‐related disease with a polygenic genetic background. The prevalence of psoriasis in China is approximately 0.47%,^1^ and is rising on a yearly basis. The subjects in this study are sourced from the Database of Chinese Center for Standardized Diagnosis and Treatment of Psoriasis. A total of 2529 psoriasis patients treated with biologics were included, of which as high as 92.37% were aged 19–60 years, and 75.19% (1,776/2,362) had moderate to severe (PASI ≥3 points) disease, constituting the majority of the patients, which is consistent with the established characteristics of the population treated with biologics for psoriasis. Psoriasis patients are typically affected by recurring conditions and generally require lifelong treatment, which brings a heavy financial burden to them, limiting the extensive use of biologics. Therefore, young and middle‐aged patients with stable income are the main user group of biologics. As China's medical insurance policy continues to improve, more people with psoriasis will assumedly have access to biologics in the future. In the present study, 24.81% of mild (PASI < 3 points) patients also opted to use biologics for treatment, which is considered to be related to the patients' pursuit of better efficacy and quality of life.

From 2009 to 2010, Chen et al.^2^ investigated 12,301 psoriasis patients in China, noting that psoriasis vulgaris was the most common (96.5%) type, of which guttate psoriasis accounted for 29.1%, while pustular psoriasis accounted for 1.6%, erythrodermic psoriasis for 0.7%, and arthritic psoriasis for 1.3%. We analyzed the psoriasis types of patients treated with biologics, noting that the highest proportion (79.79%) of patients had plaque psoriasis as the primary clinical manifestation, followed by guttate psoriasis (11.70%), erythrodermic psoriasis (3.01%), arthritic psoriasis (2.97%), localized pustular psoriasis (1.23%), and generalized pustular psoriasis (1.30%). These findings are similar to those in the investigation by Chen et al.,^2^ yet the proportion of erythrodermic psoriasis was slightly higher in the present study than in previous studies,^2^ which might be related to the fact that patients with erythrodermic psoriasis are increasingly resorting to biologics in place of conventional therapies. A number of studies have reported that biologics could provide an effective therapeutic option for erythrodermic psoriasis.^3^, ^4^ With expanding application scope of biologics, favorable therapeutic effects have also been achieved in the treatment of severe or refractory psoriasis such as arthritic and pustular psoriasis.^5^, ^6^

In comparing the use of biologics in patients with various types of psoriasis, it was noted that the highest proportion of patients used secukinumab; with the exception of patients with generalized pustular psoriasis, of which 39.39% used secukinumab, over 50% patients with all other types of psoriasis used secukinumab; adalimumab was the most commonly used biologic following secukinumab. In August 2018, the first real‐world clinical study of secukinumab in the treatment of psoriasis in China was initiated. The results suggest that the PASI75, PASI90, and PASI100 response rates to secukinumab 300 mg at 16 weeks of treatment were 95.1%, 90.1%, and 64.2%, respectively, all higher than the corresponding results of phase III clinical trials.^7^, ^8^ TNF‐α inhibitors are the earliest biologics for psoriasis approved for marketing^9^; among them, adalimumab is a fully humanized anti‐TNF‐α monoclonal antibody that has demonstrated favorable efficacy for arthritic psoriasis and plaque psoriasis.^10^ In the present study, secukinumab was the most commonly used, which might have been related to its high PASI response rate,^11^ better safety in terms of inducing infection compared with TNF‐α inhibitors,^12^ and coverage by medical insurance, etc.

In the efficacy evaluations of biologics, secukinumab had the best prior efficacy evaluation, with 93.60% of the patients being satisfied with the efficacy and only 1.23% considering it to be poor. Compared with other biologics, secukinumab not only was more commonly used, but also had a very favorable efficacy evaluation. With regard to ixekizumab, which is also an IL‐17A inhibitor, 81.03% of the patients considered it to have good efficacy; with the advancement and improvement of medical insurance policies, the proportion of patients using ixekizumab may increase.

The present study revealed varying reasons for discontinuation of biologics. Among them, the primary reason was discontinuation after disease control for secukinumab, poor efficacy for TNF‐α inhibitors, and economic reasons for ustekinumab and ixekizumab. It is noteworthy that while IL‐17 inhibitors had a good safety profile in short‐term clinical trials,^13^ in the present study, two patients were tested positive for tuberculosis and detected with hepatitis B virus replication during use of IL‐17 inhibitors; therefore, in using IL‐17 inhibitors, clinicians are expected to exercise greater vigilance and strictly follow the guidelines to regularly follow up the infection indicators, so as to minimize the development of adverse reactions/events. Other reasons of interest for discontinuation include the impact of COVID‐19, which led to drug shortage that forced the patients to interrupt treatment. In addition, no relevant data has been available yet to support the correlation between the use of biologics and the risk of contracting COVID‐19; use of biologics with downstream targets such as IL‐17 is preferred, as they would have less impact on immunity.^14^ Abdelmaksoud et al.^15^ out that for psoriasis patients currently treated with biologics, if they are tested negative for COVID‐19 or have no relevant symptoms and signs, it is not recommended to arbitrarily disrupt treatment with biologics; otherwise it may lead to the production of anti‐drug antibodies and reduced efficacy.

The present study still has some limitations. First, this study used data from the clinical big data collection platform of Chinese Center for Standardized Diagnosis and Treatment of Psoriasis for retrospective analysis, which may have led to certain selection bias. In future studies, it is desirable to broaden the sources of study subjects so that as many patients as possible could be included. Second, this study failed to investigate the reasons for drug discontinuation by patients based on statistical analysis, warranting further exploration in future studies.

Relying on the clinical big data collection platform of Chinese Center for Standardized Diagnosis and Treatment of Psoriasis, this study retrospectively analyzed the use of biologics in Chinese psoriasis patients, noting that among patients with various types of psoriasis, secukinumab was the most commonly used, and had the best patient evaluation of efficacy. The primary reason for drug discontinuation was discontinuation after disease control. These real‐world data are expected to further enrich the clinical experience of treatment with biologics, enabling clinicians to more flexibly respond to issues in using biologics for treating special types of psoriasis, and to provide data support for studies on the diagnosis and treatment of psoriasis.

## CONFLICT OF INTEREST STATEMENT

The authors declare that they have no competing interests.

## ETHICS STATEMENT

This study was conducted in accordance with the Declaration of Helsinki and approved by the ethics committee of Beijing Jishuitan Hospital (approval number: JiLunKeShenZi No.202109‐57).

Written informed consent was obtained from the participant.

## Data Availability

All data generated or analyzed during this study are included in this published article.
